This article has been retracted.

# Research on Recognition Effect of DSCN Network Structure in Hand-Drawn Sketch

**DOI:** 10.1155/2021/4056454

**Published:** 2021-11-18

**Authors:** Qunjing Ji

**Affiliations:** Graduate School, Dankook University, Yongin-si 16890, Gyeonggi-do, Republic of Korea

## Abstract

With the rapid development of image recognition technology, freehand sketch recognition has attracted more and more attention. How to achieve good recognition effect in the absence of color and texture information is the key to the development of freehand sketch recognition. Traditional nonlearning classical models are highly dependent on manual selection features. To solve this problem, a neural network sketch recognition method based on DSCN structure is proposed in this paper. Firstly, the stroke sequence of the sketch is drawn; then, the feature is extracted according to the stroke sequence combined with neural network, and the extracted image features are used as the input of the model to construct the time relationship between different image features. Through the control experiment on TU-Berlin dataset, the results show that, compared with the traditional nonlearning methods, HOG-SVM, SIFT-Fisher Vector, MKL-SVM, and FV-SP, the recognition accuracy of DSCN network is improved by 15.8%, 10.3%, 6.0%, and 2.9%, respectively. Compared with the classical deep learning model, Alex-Net, the recognition accuracy is improved by 5.6%. The above results show that the DSCN network proposed in this paper has strong ability of feature extraction and nonlinear expression and can effectively improve the recognition accuracy of hand-painted sketches after introducing the stroke order.

## 1. Introduction

With the popularization and development of Internet technology, image recognition technology began to be applied to all aspects of life [1–3]. Among them, as a common way of communication, freehand sketch has attracted more and more researchers' attention [4]. Freehand sketch recognition has become a new research hotspot in the computer field. Hand-drawn sketch is the most intuitive feeling of people for the real world [5]. It can describe the scene information with simple strokes, which has very important application significance. Compared with natural pictures, hand-painted sketches have no color and texture information, generally binary images or gray images, and have highly abstract and symbolic attributes, and there are some problems such as incomplete sketch outline due to a pause and discontinuity in the user's drawing process, which makes the recognition of hand-painted sketches a very challenging problem. At present, the basic process of hand-drawn image recognition mainly includes four steps: image preprocessing, image segmentation, image feature selection, and target recognition. The artificial selection of important parts as experimental input and the artificial selection of specified features are the main contents of image segmentation and image feature extraction respectively. They are also the key to the process of hand-drawn sketch recognition, which directly affects the final recognition effect. These methods rely heavily on manually designed feature extraction rules, which are time consuming and laborious, and different recognition results will appear due to the differences of researchers' experience and ability. Therefore, how to reduce the dependence on manual experience and achieve good recognition effect without color and texture information is an urgent problem to be solved.

With the hot development of deep learning, various deep learning models on image recognition have emerged, such as Alex-Net, VGG (Visual Geometry Group), and ResNet (Residual Network) [6–10]. Although these deep learning models avoid the artificial selection of important parts and artificial feature extraction and reduce the impact of artificial factors on the recognition effect, the design of these deep learning models is very dependent on the color and texture information of the picture, which is difficult to be directly used in the recognition of hand-painted sketches lacking color and texture information. Therefore, a neural network DSCN (Depthwise Separable Convolutions Net) based on depth separable convolution is proposed for hand-drawn sketch recognition. Firstly, the network extracts the stroke sketch sequence according to the stroke order of the hand-painted sketch, then sorts the extracted image features according to the arrangement order of the original stroke sketch, and constructs a certain time-series relationship for different image features to further improve the distinguishability of the hand-painted sketch features. Finally, the output features of the network are trained and recognized; this method avoids the unique color information of the sketch and can greatly improve the recognition of the sketch.

In order to solve the problems of lack of color and texture information, incomplete contour, large dependence on human experience, and unsatisfactory recognition effect in hand-painted sketch recognition, this paper studies and proposes a method for hand-painted sketch recognition based on DSCN network. The first section briefly introduces the background and motivation of hand-drawn sketch recognition. The second section briefly introduces the status of hand-drawn sketch recognition, discusses the problems to be solved in the current hand-drawn sketch recognition algorithm, and summarizes the work and methods of this paper. The third section first introduces the network structure based on DSCN and then gives the application process of hand-drawn sketch recognition based on DSCN model. The fourth section selects the dataset of training and testing and determines the evaluation index of model recognition effect. Then, six groups of control experiments are designed based on DSCN structure. The fifth section briefly summarizes the main conclusions of this paper.

## 2. Related Work

As the simplest and direct way of communication, hand-painted sketch can be traced back to decades ago. Due to the lack of available datasets for training and comparison, the research progress on hand-painted sketch was slow during this period. With the popularity of networks and intelligent devices, a benchmark dataset containing 250 hand-drawn sketch objects is constructed, which makes the research of hand-drawn sketch attract the attention of more and more experts and scholars.

The earlier hand-drawn sketch recognition methods followed the traditional image classification mode, that is, artificially select features and send them to the classifier for classification. Common manual features mainly include directional gradient histogram, size invariant feature transformation, and shape context feature. Qi et al. [11] proposed an improved directional gradient histogram description feature to describe the relevant features of hand-painted sketches. Hu et al. [12] used a performance evaluation of gradient field hog descriptor for sketch-based image retrieval. Chang et al. [13] used dynamic selection of shape feature points to construct contour feature point histogram. Galil et al. [14] reported a human-subject protocol study that aimed to examine cognitive chunking during freehand sketching of design ideas in engineering and correlation between chunks and the functions of the design perceived by the designer. These methods are very dependent on the extraction of artificial features. While consuming a lot of human and material resources, the recognition results are not objective and inaccurate.

With the rapid progress of computer technology, deep learning has made great progress in the field of hand-drawn sketch recognition [15–18]. Zhang et al. [19] used the sketch dataset to fine tune the parameters of a hybrid convolutional neural network and achieved good recognition results. The training ability of the first convolution layer of the neural network can be improved by using the convolution model of the first convolution layer. Li et al. [20] used deep learning model to count sketch characteristics to improve sketch recognition and similarity search. However, these methods do not consider the key feature of sketch stroke sequence, and the recognition effect of the model needs to be improved.

To sum up, although many scholars have done a lot of work in the research of hand-painted sketch recognition, the dependence of early recognition model on human feature selection and the lack of stroke sequence features of hand-painted sketch in deep learning model make the recognition effect of the model difficult to meet the expected requirements. Therefore, how to reduce the dependence on human experience and consider more image features is of great significance in the field of hand-drawn sketch recognition. In view of this, this paper uses DSCN network for hand-drawn sketch recognition. The model uses the stroke timing information of hand-drawn sketch to improve the recognition accuracy of the model and has a good recognition effect.

## 3. Hand-Drawn Sketch Recognition Based on DSCN Network Structure

### 3.1. Neural Network Model of DSCN Network Structure

Convolution is a very important mathematical operation in artificial neural network [21–24]. It can successfully avoid the dependence of traditional networks on manual feature selection and has been widely used in the field of image recognition. Convolutional neural networks (CNNs) are a kind of feedforward neural networks with depth structure including convolution calculation. It is one of the representative algorithms of depth learning [25–32]. Convolution neural network imitates the visual perception mechanism of biology, which can carry out supervised learning and unsupervised learning. The essence of convolutional neural network is a multilayer perceptron, which contains many neurons and is composed of input layer, hidden layer, and output layer. The input layer inputs feature points represented by each pixel. The convolution layer and convergence layer of the hidden layer are the core of image feature extraction. The overall network structure is shown in Figure 1.

In the image convolution operation, each neuron convolutes and sums the image matrix input from the previous layer with the convolution cores of multiple large and small pen holders, followed by an additive bias, solves the additive bias and multiplicative bias as the parameters of the excitation function, and outputs a new value after the linear rectification function activation, so as to form a new characteristic image. In the convolution process of a standard convolution neural network, *x*_11_, *x*_12_,…, *x*_44_ is the pixel value of the input image, *ω*_11_, *ω*_12_,…, *ω*_44_ is the weight of the convolution kernel, and *y*_11_, *y*_12_,…, *y*_44_ is the characteristic image obtained after convolution. Then the pixel value of the output image is

(1) $$\begin{array}{c} y_{ij}=\sum_{i=1}^{3}\sum_{j=1}^{3}\omega_{ij}x_{ij}. \end{array}$$

There are two important parameters in convolution operation: the size of convolution kernel and sliding step size. The size of the convolution kernel determines the size of the receptive field and the interval pixels of each sliding of the step giant top. In addition, filling is also a parameter of the convolution layer, assuming that the input image is *M* × *M*. The convolution kernel size is *K* × *K*. The step size is *S*, the filling is *P*, and the output feature image size is *N* × *N*. Then *N* is expressed as

(2) $$\begin{array}{c} N=\frac{M-K+2P}{S}+1. \end{array}$$

The output of each neuron in the convolution layer is

(3) $$\begin{array}{c} Y_{j}^{L}=f\left(\sum_{i=1}^{N^{L-1}}Y_{i}^{L-1}⊗w_{ij}^{L}+b_{j}^{L}\right). \end{array}$$

In formula (3): *L* and *L* − 1 are the depth of the network layer; *f*() is the activation function; ⊗ represents convolution operation; *Y*_*j*_^*L*^ represents the *j*-th output characteristic image of the *L*-th layer; *Y*_*i*_^*L*−1^ represents the characteristic image output from layer *L* − 1; *w*_*ij*_^*L*^ and *b*_*j*_^*L*^ represent the multiplicative bias and additive bias of *L* layer, respectively.

As shown in Figure 2, the depth separable convolution proposes an idea of processing the image corresponding region and channel separately, first considering the region features and then considering the channel features. Different from the traditional convolution, considering all channels at the same time, the depth separable convolution operation can be decomposed into two processes: depthwise and pointwise. Compared with ordinary convolution calculation, the compression *P* of depth separable convolution calculation is shown in

(4) $$\begin{array}{c} P=\frac{\text{depthwise}+\text{pointwise}}{\text{convolution}}\\ =\frac{H\times W\times C\times n\times n+H\times W\times C\times k}{H\times W\times C\times k\times n\times n}=\frac{1}{k}+\frac{1}{n\times n}\approx \frac{1}{n\times n}. \end{array}$$

In equation (4), the input image pixel is *N* × *H* × *W* × *C*; the size of convolution kernel is *n* × *n* × *k*; the output is *N* × *H* × *W* × *C*. The calculated compression amount P is similar to (1/(*n* × *n*)); that is, compared with the ordinary convolution operation, the operation based on deep separable convolution can greatly reduce the amount of convolution calculation.

Pooling is another frequently used operation in convolutional neural network. Its main function is to downsample the image to obtain more effective information. The pooling operation is generally divided into average pooling and maximum pooling. Average pooling takes the average value of the pooling area as the output, and its calculation formula is

(5) $$\begin{array}{c} y_{11}=\frac{x_{11}+x_{12}+x_{13}+x_{14}}{4}. \end{array}$$

Maximum pooling is to take one of the maximum values as the pooling result, and its calculation formula is

(6) $$\begin{array}{c} z_{11}=\max\left(x_{11},x_{12},x_{21},x_{22}\right). \end{array}$$

In equations (5) and (6), *x*_11_, *x*_12_,…, *x*_44_ is the pixel value of the input image and *y*_11_, *y*_12_,…, *y*_22_ is the average pooling result; *z*_11_, *z*_12_,…, *z*_22_ is the maximum pool result. The difference between pooling operation and convolution operation is that pooling operation has a convolution kernel with parameters that can be learned, while pooling operation only operates according to the rule of finding the mean or maximum value. When the convolution neural network is in convolution layer, pool layer, and full-connection layer, it needs to calculate the loss through loss function. The commonly used loss functions include square loss function and cross entropy loss function. For a sample, the square loss function is expressed as follows:

(7) $$\begin{array}{c} E=\frac{1}{2}\sum_{i=1}^{k}{\left(a_{i}^{L}-y_{i}\right)}^{2}=\frac{1}{2}{\left\|a^{L}-y\right\|}^{2}. \end{array}$$

In equation (7), *a*_*i*_^*L*^ is the *i*-th element of *a*^*L*^, which is the network output unit; *y*_*i*_ is the *i*-th element of *y*, and *y* is the label vector. The calculation result of convolution operation in the forward propagation of data in convolution neural network can be expressed as

(8) $$\begin{array}{c} F^{l}=\text{conv}\left(a^{l-1}\right)=\sum_{k=1}^{M}\left(a_{k}^{l-1}*W_{k}^{l}\right)+b^{l}. \end{array}$$

In equation (8), conv(·) represents the convolution operation, *F*^*l*^ is the output of the convolution operation, *W*_*k*_^*l*^ is the weight matrix of the *k*-th output characteristic graph corresponding to the *L*-th layer, *∗* is the convolution operation, and *b*^*l*^ is the offset of the *l*-th layer. An activation function will be connected behind the convolution layer to increase the nonlinearity of the network. As the most widely used activation function, the expression of RrLU is

(9) $$\begin{array}{c} y=\left\{\begin{array}{cc} x, & x\geq 0,\\ 0, & x<0. \end{array}\right. \end{array}$$

The derivative function expression of RrLU activation function is

(10) $$\begin{array}{c} y=\left\{\begin{array}{cc} 1, & x\geq 0,\\ 0, & x<0. \end{array}\right. \end{array}$$

If act(·) represents the activation function, the output result of the activation function is

(11) $$\begin{array}{c} a^{l}=\text{act}\left(F^{l}\right)=\text{act}\left(\text{conv}\left(a^{l-1}\right)\right)=\text{act}\left(\sum_{k=1}^{M}\left(a_{k}^{l-1}*W_{k}^{l}\right)+b^{l}\right). \end{array}$$

Pooling layer operations can be expressed as

(12) $$\begin{array}{c} a^{l}=\text{pool}\left(a^{l-1}\right). \end{array}$$

In equation (12), pool(·) is the pool operation, *a*^*l*^ is the output of the pool layer, and *a*^*l*−1^ is the input of the pool layer. The calculation process of data forward propagation to the full-connection layer is as follows:

(13) $$\begin{array}{c} a^{l}=\text{act}\left(F^{l}\right)=\text{act}\left(\text{fc}\left(a^{l-1}\right)\right)=\text{act}\left(W^{l}a^{l-1}+b^{l}\right). \end{array}$$

In equation (13), *a*^*l*−1^ is the input of the full-connection layer, fc(·) is the full-connection operation, *F*^*l*^ is the output of the full-connection layer, and *a*^*l*^ is the output after activating the function. Convolutional neural networks are mostly composed of convolution layer, pool layer, and full-connection layer. Equations (7)∼(13) show the general process of forward propagation of convolutional neural networks.

### 3.2. Hand-Drawn Sketch Recognition Based on DSCN Network Structure Model

This paper proposes an end-to-end hand-drawn sketch recognition network based on DSCN, which can perform accurate detection and recognition tasks and has good recognition effect for hand-drawn sketches. Its network structure is divided into encoder and decoder, mainly including five modules: input, standard volume module, depth separable convolution module, deconvolution module, and output, as shown in Figure 3(a).

Hand-drawn sketch recognition based on depth separable convolution neural network is mainly divided into two stages: model training and testing, as shown in Figure 3(b). In the training stage, a fixed number of images are randomly selected from the training hand-painted sketch samples as the input of the DSCN neural network model, and then the predicted value of the hand-painted sketch category is output through the model, and then the backpropagation gradient is calculated by the loss function to update the network parameters.

As can be seen from Figure 3, the network is mainly composed of encoder decoder structure. Encoder decoder refers to a device or program that can transform a signal or a data stream. The encoder part needs to set the width multiplier and resolution multiplier to weigh the parameter scale, running speed, and recognition accuracy of the whole network. The decoding part is composed of deconvolution module and depth separable module. The convolution kernel size of all deconvolution operations is 2 × 2, and step size is 2.

In the network training, the random gradient descent algorithm is used as the parameter optimizer; the learning rate is 0.001, the momentum is 0.9, and the training batch is 16. When single channel labeling information is input into network training, the activation function of the last layer is sigmoid, which is defined as

(14) $$\begin{array}{c} y\left(x\right)=\frac{1}{1+e^{\alpha \left(x\right)}}. \end{array}$$

In equation (14), *α*(*x*) represents the output value predicted by pixel *x* on the image for a certain category and *y*(*x*) is the probability that pixel *x* on the image belongs to this category. The loss function is the opposite number of DICE coefficients, defined as

(15) $$\begin{array}{c} L=-\frac{2\times \left|y_{\text{true}}\cap y_{\text{pred}}\right|}{\left|y_{\text{true}}\right|+\left|y_{\text{pred}}\right|}. \end{array}$$

In equation (15), *y*_true_ represents the normalized single category annotation image and *y*_pred_ represents the prediction image input by the sigmoid layer.

## 4. Research on Hand-Drawn Sketch Recognition Effect Based on DSCN Network Model

### 4.1. TU-Berlin Dataset and Evaluation Indicators

TU-Berlin dataset is a challenging benchmark dataset in the task of hand-drawn sketch recognition and classification. It includes 250 different categories of objects, and the original pixel size of the sketch is 1111 × 1111. Four-fold cross validation was used in the experimental process, 3 for training and 1 for testing. An example sketch is shown in Figure 4.

In order to study the influence of dataset size on training recognition accuracy, we divide the dataset into 8, 16, 24,…, 80 sketches in each category, a total of 10 datasets of different sizes. Using the four methods of KNN hard, KNN soft, SVM hard, and SVM soft given by Eitz, the average cross validation accuracy of these subdatasets is three times. Therefore, in order to prevent the overfitting problem caused by the lack of training data in the training process, the existing dataset is manually expanded by dimensionality reduction, slice extraction, horizontal flip, and other operations.

The average accuracy MAP (Mean Average Precision) is selected as the evaluation index of the evaluation model in the hand-drawn sketch recognition task, and the average accuracy MAP can be expressed as

(16) $$\begin{array}{c} \text{MAP}=\frac{1}{N}\sum_{1}^{N}\frac{m}{n}. \end{array}$$

In equation (16), *m* is the number of hand-drawn sketches correctly identified, and *n* is the total number of test data of a category.

### 4.2. Recognition Effect of Different Network Hand-Drawn Sketches

In order to test the recognition effect of DSCN network structure in hand-drawn sketches, six groups of comparative experiments are designed in this paper. In the first group of experiments, the CNN neural network based on standard convolution is compared with the DSCN network model based on depth separability proposed in this paper, and the recognition accuracy is compared on the original dataset. The experimental results are shown in Figure 5.

As can be seen from Figure 6, DSCN network based on deep separable convolution has stronger recognition ability than CNN network based on standard convolution. In addition, with the introduction of sketch stroke order and the increase of training dataset, the recognition effect of the model will be enhanced.

The second group of experiments discussed the influence of the number of extracted substroke sketches on the recognition accuracy. Experiments were carried out on 2 substroke sketches, 3 substroke sketches, and 4 substroke sketches extracted from each sketch image. The experiments were carried out on the expanded dataset. The experimental results are shown in Figure 6.

Figure 6 shows the influence of the number of extracted substroke sketches on the recognition accuracy. In these five groups of comparative experiments, the recognition accuracy of extracting 3 substroke sketches is higher than that of extracting 2 substroke sketches and 4 substroke sketches. The experimental results show that when the number of extracted substroke sketches is too small, the stroke order information is too small. When too many substroke sketches are extracted, too much stroke order information is introduced, which will overfit the stroke order of the detail part of the painting, resulting in the decline of recognition accuracy. In addition, it can be seen that the model achieves the best recognition effect when the number of hidden layer neurons is 2000.

The third group of experiments discusses the influence of the variance *σ* of initialization connection weights *ω*_*ih*_ and *ω*_*hh*_ on the recognition accuracy in the DSCN network model. The experimental results are shown in Figure 7.

Figure 7 shows the influence of variance *σ* of initialization weights *ω*_*ih*_ and *ω*_*hh*_ in DSCN network on recognition accuracy. The experimental results show that when *σ*=0.02, the recognition accuracy is slightly better than when the variance *σ* is 0.01 and 0.03. This is because when the variance is too small, the value range of the weight is small, which easily leads to the small value difference of the elements in the feature expression vector of the hidden layer, reducing the resolution of the feature vector. When the variance is too large, it is easy to lead to the value of too many elements in the eigenvector close to 0 or 1, which will also reduce the separable deformation of the eigenvector. The three groups of variance achieved the best recognition accuracy when the hidden layer reached 2000, which were 71.62%, 71, 80%, and 71.72%, respectively.

In order to clarify the impact of sampling points on recognition performance, the fourth group of experiments quantitatively analyzed the sampling points. At the same time, for better comparative experiments, sketchy dataset was introduced. The experimental results are shown in Figure 8.

As can be seen from Figure 9, with the increase of sketch points, the accuracy of model recognition is also improving. When the points are close to 1000, the accuracy reaches saturation. At this time, continue to increase points, and the accuracy will decline. The reason for this phenomenon is that too many points will make the local pattern repeat, which will affect the representation of discriminant features, so as to reduce the accuracy of recognition.

In order to prove the advantages of DSCN network, the fifth group of experiments selected some difficult cases on TU-Berlin dataset for identification and comparison. The experimental results are shown in Figure 9.

As can be seen from Figure 9, compared with the DNN neural network of standard convolution, the DSCN network based on deep separable convolution has better performance in identifying some difficult cases. Finally, DSCN network is compared with other mainstream hand-drawn sketch recognition algorithms such as HOG-SVM, SIFT-Fisher Vector, MKL-SVM, FV-SP, and Alex-Net. The experimental results are shown in Figure 10.

As can be seen from Figure 10, compared with the traditional nonlearning methods, HOG-SVM, SIFT-Fisher Vector, MKL-SVM, and FV-SP, the recognition accuracy of DSCN network is improved by 15.8%, 10.3%, 6.0%, and 2.9%, respectively. The results show that this method has stronger depth learning ability and nonlinear feature extraction ability. Compared with the classical deep learning model Alex-Net, the recognition accuracy is improved by 5.6%. The results show that the introduction of stroke order in hand-drawn sketch can effectively improve its recognition accuracy.

## 5. Conclusion

In view of the dependence of traditional nonlearning classical model on manually selected features and the dependence of deep learning model on color and texture information in hand-drawn sketch recognition, a neural-network-based hand-drawn sketch recognition method based on DSCN structure is proposed in this paper. The model considers the stroke sequence information of hand-drawn sketch and has strong ability of feature extraction and nonlinear expression. Through the control experiment on TU-Berlin dataset, the results show that compared with the traditional nonlearning methods, HOG-SVM, SIFT-Fisher Vector, MKL-SVM, and FV-SP, the recognition accuracy of DSCN network is improved by 15.8%, 10.3%, 6.0%, and 2.9%, respectively. Compared with the classical deep learning model Alex-Net, the recognition accuracy is improved by 5.6%. The above results show that the DSCN network structure proposed in this paper performs well in the field of hand-drawn sketch recognition and provides a new method for hand-drawn sketch recognition. However, the research of this paper does not carry out detailed data simulation of sketch recognition algorithm, which makes the practical application of the research have a certain swing. Therefore, it needs to be supplemented in future research.

## Figures and Tables

**Figure 1:** General structure of hidden layer in deep convolution neural network.

**Figure 2:** Depth separable convolution: depthwise convolution process and pointwise convolution process.

**Figure 3:** Construction of network structure model and training process of hand-drawn sketch recognition based on DSCN. (a) Deep separable convolutional neural network structure. (b) Flow chart of hand-drawn sketch recognition based on DSCN network structure.

**Figure 4:** TU-Berlin dataset sample image.

**Figure 5:** Comparison of recognition accuracy between DSCN and CNN on different Tu-Berlin datasets.

**Figure 6:** Influence of the number of substroke sketches on recognition accuracy.

**Figure 7:** Influence of initialization variance on recognition accuracy.

**Figure 8:** Influence of different sampling points on recognition accuracy.

**Figure 9:** Recognition accuracy of some difficult cases on Tu-Berlin dataset.

**Figure 10:** Comparison of recognition effect between DSCN model and existing recognition methods.

## Data Availability

The data used to support the findings of this study are available from the corresponding author upon request.
